# The Need for Improved Identification and Accurate Classification of Stages 3–5 Chronic Kidney Disease in Primary Care: Retrospective Cohort Study

**DOI:** 10.1371/journal.pone.0100831

**Published:** 2014-08-12

**Authors:** Poorva Jain, Melanie Calvert, Paul Cockwell, Richard J. McManus

**Affiliations:** 1 Primary Care Clinical Sciences, NIHR School of Primary Care Research, University of Birmingham, Birmingham, United Kingdom; 2 Department of Renal Medicine, Queen Elizabeth Hospital Birmingham, University Hospital Birmingham, Birmingham, United Kingdom; 3 Division of Immunity and Infection, Medical School, University of Birmingham, Birmingham, United Kingdom; 4 Department of Primary Care Health Sciences, NIHR School of Primary Care Research, University of Oxford, Oxford, United Kingdom; University of South Florida, United States of America

## Abstract

**Background:**

Around ten percent of the population have been reported as having Chronic Kidney Disease (CKD), which is associated with increased cardiovascular mortality. Few previous studies have ascertained the chronicity of CKD. In the UK, a payment for performance (P4P) initiative incentivizes CKD (stages 3–5) recognition and management in primary care, but the impact of this has not been assessed.

**Methods and Findings:**

Using data from 426 primary care practices (population 2,707,130), the age standardised prevalence of stages 3–5 CKD was identified using two consecutive estimated Glomerular Filtration Rates (eGFRs) seven days apart. Additionally the accuracy of practice CKD registers and the relationship between accurate identification of CKD and the achievement of P4P indicators was determined. Between 2005 and 2009, the prevalence of stages 3–5 CKD increased from 0.3% to 3.9%. In 2009, 30,440 patients (1.1% unadjusted) fulfilled biochemical criteria for CKD but were not on a practice CKD register (uncoded CKD) and 60,705 patients (2.2% unadjusted) were included on a practice CKD register but did not fulfil biochemical criteria (miscoded CKD). For patients with confirmed CKD, inclusion in a practice register was associated with increasing age, male sex, diabetes, hypertension, cardiovascular disease and increasing CKD stage (p<0.0001). Uncoded CKD patients compared to miscoded patients were less likely to achieve performance indicators for blood pressure (OR 0.84, 95% CI 0.82–0.86 p<0.001) or recorded albumin-creatinine ratio (OR 0.73, 0.70–0.76, p<0.001).

**Conclusions:**

The prevalence of stages 3–5 CKD, using two laboratory reported eGFRs, was lower than estimates from previous studies. Clinically significant discrepancies were identified between biochemically defined CKD and appearance on practice registers, with misclassification associated with sub-optimal care for some people with CKD.

## Introduction

Chronic Kidney Disease (CKD) is defined by a reduced glomerular filtration rate (GFR) and/or evidence of kidney damage and in clinical practice a reduced eGFR is usually estimated using the Modification of Diet in Renal Disease (MDRD) four-variable equation [1]. Patients with an eGFR below 60 mls/min/1.73 m^2^ (stages 3–5 CKD) are at increased risk of cardiovascular disease (CVD), in comparison to the general population [2]–[4]. Between 2009–2010, CKD accounted for 1.3% of the UK health care budget directly and indirectly up to 25% of the healthcare budget in the United States in patients aged over 65 [5], [6]. In the past decade there have been sustained efforts to improve the identification, management and monitoring of CKD [7]. In the UK this has included the incorporation of stages 3–5 CKD into the Quality and Outcomes Framework (QOF), a primary care based pay for performance system (P4P) [8], [9]. Incentivised payments within the CKD domain depend on blood pressure control and appropriate prescribing [10].

Previous estimates of the prevalence of stages 3–5 CKD have varied widely (depending on the methodology) from 4.3% (all clinically coded patients in QOF) to 8.5% in UK primary care databases [11]. Potential sources of bias include ascertainment problems (reliance on coding, limited coverage of population), intra patient variation in renal function (single eGFR likely to overestimate prevalence) and intra-laboratory variation (use of raw creatinines to calculate eGFR does not take into account calibration issues between labs) [12]. Accurate identification and subsequent clinical coding of CKD is important, as previous work suggests that inclusion on a chronic disease register affects quality of care [13].

This study aimed to determine the prevalence of stages 3–5 CKD based on objective evidence from at least two laboratory reported eGFRs and to assess the accuracy of QOF CKD (stages 3–5) registers on this basis. The quality of care for patients with stages 3–5 CKD was compared between those who were included on a CKD register and those who had laboratory evidence of stages 3–5 CKD but were not included on a register.

## Materials and Methods

### Data source

A retrospective cohort study was undertaken using anonymised records from The Health Improvement Network (THIN) database. In brief this is a large UK primary care database that contains data from patients registered in 426 primary care centres using VISION clinical software; in 2009 2.7 million patients were included [14]. The THIN database has previously been validated for use in pharmaco-epidemiological research [14], [15]. Permission to obtain and analyse this data has to be sought from the THIN Scientific Review Committee and was granted for our study in May 2010 (reference number 10-006).

Data were extracted from the THIN database concerning renal function, age (on 1^st^ April of the year of the prevalence estimate), registration status, gender, Read codes indicating co-morbidity (cardiovascular disease, diabetes, hypertension, chronic kidney disease, and hypercholesterolemia) and cardiovascular risk factors (smoking status, blood pressure, ACR and total cholesterol). Read codes are a system of hierarchal clinical codes that specify types of diseases, symptoms, diagnoses or other medical information from consultations or letters. Co-morbidities were defined using previously described code groupings and the authors' clinical expertise [16], [17].

### Prevalence: study population

Adults with stages 3–5 CKD, permanently registered on the THIN database for a minimum of six months, were identified if the last two laboratory eGFRs in each UK financial year (April – March) between 2005 and 2009, taken at least seven days apart, were both <60 ml/min/1.73 m^2^ (Figure 1). This definition was used as a pragmatic operationalization of UK pay for performance (QOF) guidance which states that stages 3–5 CKD is defined as an eGFR <60 mls/min/1.73 m^2^ “…confirmed with at least two separate readings over a three month period”. Note this is different to the KDIGO/KDOQI definition of CKD [7], [18]. Ethnicity data were not available for the large majority of patients who were therefore assumed to be not of black ethnicity [19].

**Figure 1:** The definition of Stages 3–5 CKD in the prevalence cohort.

Patients identified as having CKD in a given year could be reclassified in following years if their eGFRs changed. Where two laboratory eGFRs were in different CKD stages, the lowest corresponding CKD stage was used; i.e. the more conservative estimate. Patients with a laboratory biochemical definition of stages 3 -5 CKD were defined as having confirmed CKD (Figure 1) for use in the subsequent QOF CKD disease register analysis. In common with previous work, people without a kidney function measurement were assumed not to have CKD [20].

### QOF outcomes: population

This analysis considered QOF performance between April 2008 and March 2009 and included risk factor data from January 2008. Stages 3–5 CKD was defined on the basis of laboratory eGFRs, to avoid issues with laboratory to laboratory variation and assuming that practices had not calculated eGFR themselves. Appearance on practice CKD registers was defined by a relevant clinical (Read) code specified by the UK pay for performance, QOF business rules which include only patients with stages 3–5 CKD [16]. On this basis, patients were categorised as having either ‘confirmed CKD’ or ‘labelled CKD’ dependent on biochemical evidence and/or Read coding. These were further divided into subgroups of ‘appropriately coded’ CKD patients, ‘uncoded CKD patients’ or ‘miscoded CKD patients’ as defined below.

- **Confirmed CKD:** sustained biochemical evidence of stages 3–5 CKD, i.e. a laboratory eGFR under 60 mls/min/1.73 m^2^ on the last two consecutive eGFRs before 1^st^ April 2009 that were at least seven days apart.
- **Labelled CKD:** patients recorded as having stages 3–5 CKD by a Read code according to the UK pay for performance (QOF) Business Rules [10], [21].
- **Appropriately coded:** patients with both a Read Code for CKD and biochemical evidence of an eGFR under 60 mls/min/1.73 m^3^ on the last two consecutive eGFRs before 1^st^ April 2009 that were at least seven days apart.
- **Uncoded CKD:** patients with biochemical evidence of stages 3–5 CKD but no CKD Read code entered into their records.
- **Miscoded CKD:** patients with a Read code for stages 3–5 CKD but no biochemical evidence of stages 3–5 CKD (using above definition).

### Statistical analyses

The prevalence of CKD was ascertained and tabulated by stage and year for the years 2005–2009. Prevalence estimates were age standardised using the relevant Office of National Statistics yearly estimates of age and gender distribution for the United Kingdom and 95% confidence intervals were calculated [22]. The management of each subgroup according to the CKD indicators of the QOF for the period of 1^st^ January 2008 and 1^st^ of April 2009 was evaluated [16].

Factors associated with the likelihood of being excluded from the practice CKD register were analysed in two subgroups:

- uncoded compared to appropriately coded
- uncoded compared to miscoded

These subgroups were examined in two multivariable models using backward stepwise selection (α = 0.05 as criteria for model inclusion). Multivariable models allow a series of factors to be assessed simultaneously to take into account possible confounding. Non-linear functional forms were considered for continuous candidate variables. More complex functional forms were included in the final model only when they provided a statistically significantly improved model fit assessed using Akaike's Information Criterion [23]. The final model included the selected variables in a mixed linear model with logit link and with general practice as a random effect to account for clustering [24], [25].

The following pre-specified explanatory variables were included in the backwards selection process: age, gender, Townsend quintiles, coronary heart disease, stroke, peripheral vascular disease, cardiovascular disease (coronary heart disease, stroke, peripheral vascular disease combined), hypertension, diabetes mellitus, smoking status and hypercholesterolaemia.

Achievement for each quality indicator was compared between miscoded and uncoded CKD patients using Pearson Chi-Square tests. Blood pressure and cholesterol comparisons were carried out using t-tests or Mann Whitney tests depending on the distribution of the variable.

All statistical analyses were performed in SAS v9.2 (Cary, USA).

### Sensitivity Analysis

A separate sensitivity analysis ascertained the prevalence of stage 3–5 CKD from the last two consecutive creatinines, taken at least 7 days apart, utilising the four variable MDRD equation to calculate the eGFR, when laboratory eGFRs were not available [26]. This analysis was undertaken as it was anticipated that prior to 2007 many patients would not have reported laboratory eGFR. The standardised Isotope Dilution Mass Spectrometry (IDMS) method for creatinine measurement was in use in less than 50% of UK laboratories during the study timeframe hence it was assumed that this method had not been used [12].

## Results

Results were adjusted for age and gender where possible but are presented as crude proportions where this is not stated.

### Prevalence of Chronic Kidney Disease

Between 2005 and 2009, the number of patients with two lab eGFRs, at least seven days apart, in the given year increased from 53 176(2%) to 614 590 (23%). The median time apart from each laboratory report in our study was 171 days (Interquartile range 56–351 days) and by 2009 this was 280 days (125–425 days). The age and gender adjusted prevalence of stages 3–5 CKD increased from 0.28% (95% CI 0.28 to 0.29) to 3.93% (3.91 to 3.95) between 2005 and 2009 (Figure 2). The majority of patients had stage 3a CKD with an adjusted prevalence in 2009 of 2.86% (2.84 to 2.87), followed by stage 3b CKD (0.86%, 0.86 to 0.87), stage 4 CKD (0.18%, 0.176 to 0.184) and stage 5 CKD (0.03, CI 0.28 to 0.03).

**Figure 2:** Age standardised prevalence (%) of stages 3–5 CKD from 2005–2009. CKD stage was defined by the last two consecutive laboratory eGFRS at least seven days apart in the year in question. Note figures are approximated to the nearest decimal place and therefore may be slightly different from the total figure.

### Practice Registers of CKD

In 2009, 108 911/2 701 730 (4.03% 95% CI 4.01–4.05) of the adult population had biochemically confirmed chronic kidney disease (see methods for definitions) and 139 176 (5.15%, 95% CI 5.13–5.18) appeared on practice registers (labelled CKD) [Table 1]. Of those with biochemically confirmed CKD, 78 471/108 911 (72.1%, 95% CI 71.8–72.3) were labelled with a Read code for stages 3–5 CKD. A further 60 705/139 176 (43.6%, 95% CI 43.3–43.9) of labelled CKD patients had a Read code but no biochemical evidence of stages 3–5 CKD (i.e. were miscoded) and 30 440/108 911 (27.9%, 95% CI 27.7–28.2%) fulfilled biochemical criteria for stages 3–5 CKD but were not on a practice CKD register (uncoded CKD). The demographic and clinical features are shown in Table 1.

**Table 1:** Demographics of CKD patients between 1st January 2008 to 1st April 2009 (The proportions in brackets are not adjusted and crude percentages).

	Total Population	Patients with biochemical evidence of CKD^a^	Practice CKD Register (with or without biochemical evidence)^b^	Patients on CKD register with biochemical evidence^c^	Practice CKD Register but no biochemical evidence of Stages 3–5 CKD^d^	Patients with biochemical evidence of CKD not on Practice Register^e^
True CKD status	Baseline Population	Confirmed CKD	Labelled CKD	Appropriately coded CKD	Miscoded CKD	Uncoded CKD
Number (crude %)	2 707 130 (100)	108 911 (4.0%)	139 176 (5.1%)	78 471 (2.9%))	60 705 (2.2%)	30 440 (1.1%)
Age in years (median (IQR))	47(19–114)	79(19–106)	76 (19–106)	78 (19–106)	71(19–105)	76(19–105)
Female Gender	1378 422(51%)	67 352 (62%)	82 949 (60%)	47 666(60%)	35 283 (58%)	19 686 (65%)
Ethnic Group^f^						
Black	11 329(0.40%)	528 (0.48%)	592(0.43%)	324(0.41%)	268(0.44%)	204(0.67%)
White	355 121(13%)	25 381 (23%)	29 820(21.4%)	18 764(23%)	11 056(18%)	6617(21%)
South Asian	20 032(0.70%)	594 (0.54%)	1051(0.76%)	468(0.59%)	583(0.96%)	126(0.41%)
Diabetes Mellitus^g^ ^f^	174 622(6%)	26 985 (25%)	33 083(23%)	20 970(26%)	12 113(20%)	6015(19%)
Hypertension	413 235(16%)	63 917(59%)	73 037(52%)	48 587(62%)	24 450(40%)	15 330 (50%)
CHD^g^ ^f^	158 701(6%)	31 234(29%)	35 471(25%)	24 254(30.8%)	11 217(18%)	6980(23%)
PVD^g^ ^f^	35 033(1%)	8330(8%)	9011(6%)	6656(8.5%)	2355(4%)	1674(5.5%)
Stroke^g^ ^f^	67 075(3%)	14 339((13%)	15 370(11%)	11 020(13.9%)	4350(7%)	3319(11%)
Ever Smoked	446 034(17%)	20 805(19%)	24 301(17%)	15 296(19%)	9005(15%)	5509(18%)

a Patients with two consecutive eGFRS under 60 at least seven days apart.

b Patients with a QOF business Rule Read code for Chronic Kidney Disease.

c Patients with 2 consecutive eGFRS <60 at least 7 days apart and a QOF business rule Read code.

d Patients with a QOF business Rule Read code for CKD but no sustained eGFRs below 60.

e Patients with 2 consecutive eGFRS <60 at least 7 days apart but no QOF Read code for CKD.

f Where reported as not all patients have Ethnic group reported.

g Diabetes Mellitus – Type 1&2, CHD = Coronary Heart Disease, PVD = peripheral vascular disease.

### Multivariable analysis

In the multivariable analyses, uncoded CKD patients in comparison with appropriately coded patients were more likely to be younger (for an increase in one year of age OR 0.991, 95% CI 0.989–0.993), female (OR 1.20, 95% CI 1.16–1.25), have no comorbidity and have a lower CKD stage [Table 2].

**Table 2:** Multivariate Logistic Regression Model for significant predictors for inclusion on CKD QOF register.

Risk Factor	Odds Ratio of Uncoded CKD compared to appropriately Coded CKD	Odds Ratio of Uncoded CKD compared to miscoded CKD
	Odds Ratio (95% CI)	Odds Ratio (95% CI)
Age^I^	0.991(0.990–0.993)	1.027(1.026–1.028)*
Female sex^II^	1.20(1.16–1.24)	1.23(1.17–1.26)*
CKD stage		NA
3aIII	1*	
3b	0.37(0.35–0.38)	
4	0.24(0.22–0.27)	
5	0.24(0.19–0.31)	
Coronary Heart Disease^iv^	0.81(0.76–0.86)*	0.80(0.74–0.86)*
Hypertension^iv^	0.61(0.59–0.63)*	1.11(1.02–1.15)*
Diabetes Mellitus	0.72(0.69–0.75)*	0.84(0.77–0.89)*
Cardiovascular Disease(composite of Coronary Heart Disease, Peripheral Vascular Disease and Stroke)	0.83(0.78–0.88)*	1.21(1.13–1.30)*
Peripheral Vascular Disease^iv^	0.88(0.82–0.95)*	NS
Hypercholesterolaemia^iv^	0.80(0.76–0.84)*	0.90(0.84–0.97)*
Smoking^iv^	NS	1.21(1.16–1.30)*

*p<0.0001.

i For an increase in years from the mean age.

ii In comparison with male gender.

iii Indicates the reference indicator.

iv The presence of the disease in comparison to those without it. The disease was ascertained by having a Read code for the disease.

In the second model uncoded patients were more likely to be older (for every year increase, OR 1.027, 95% CI 1.026–1.208), have hypertension (OR 1.11, 95% CI 1.02–1.15), cardiovascular disease (OR 1.21, 95% CI 1.13–1.30), and to smoke (OR 1.21, 95% CI 1.16–1.30) compared to miscoded patients. They were less likely to have diabetes (OR 0.84, 95% CI 0.77–0.89), coronary heart disease (OR 0.80, 95% CI 0.74–0.86), and have hypercholesterolaemia (OR 0.90, 95% CI 0.84–0.97) [Table 2].

### Pay for Performance

The management of CKD patients according to QOF P4P indicators is shown in Table 3. There was significant underachievement in QOF outcomes in the uncoded CKD group compared to both the miscoded CKD group and the appropriately coded CKD group: uncoded CKD patients were less likely to have a blood pressure measurement (90% versus 91% in miscoded group, p<0.0001, 90% vs. 97% in appropriately coded group, p<0.0001), a blood pressure on target (47% vs. 51%, p<0.0001, 47% vs. 55%, p<0.0001). or have an albumin-creatinine ratio recorded (12% vs. 16%, p<0.0001, 12% vs. 20%, p<0.0001). Mean systolic blood pressure, in mmHg, was significantly higher in patients with uncoded CKD [136.2 (95% CI 136.0 to 136.4)/75.8 (75.7 to 75.9) compared to miscoded CKD 134.5 (134.3 to 134.6)/76.3 (75.0 to 75.1)]. Cholesterol was measured in 92% of individuals regardless of group. There was no difference in serum cholesterol level between miscoded and uncoded CKD (median cholesterol 4.7 vs. 4.7 mmol/l, p = 0.9455). All patients with proteinuria as defined by an ACR ≥30 mg/mmol and with a Read code for hypertension (n = 1018) were on angiotensin blockade regardless of CKD coding [Table 3].

**Table 3:** CKD Management according to QOF standards between 1st January 2008 to 1st April 2009+.

	Patients with biochemical evidence of CKD^a^	Practice CKD Register(with or without biochemical evidence)^b^	Patients on CKD register with biochemical evidence^c^	Practice CKD Register but no biochemical evidence of Stages 3–5 CKD^d^	Patients with biochemical evidence of CKD not on Practice Register^e^
True CKD status	Confirmed CKD	Labelled CKD	Appropriately coded CKD	Miscoded CKD	Uncoded CKD
Total Number	108 911	139 176	78 471	60 705	30 440
Proportion with Blood pressure in last 15 months*	104 213(96%)	132 343(95%)	76 602(97%)	55 741(91%)	27 611(90%)
Patients whose last BP is less than 140/85 in last 15 months*	57 169(52%)	73 852(53%)	42 986(55%)	30 866(51%)	14 183(47%)
Patients with CKD who have an ACR*	19 483(18%)	25 445(18%)	15 806(20%)	9639(16%)	3677(12%)
Patients with CKD who have Proteinuria *	1358(1.2%)	1474(0.9%)	1153(1.4%)	320(0.5%)	205(0.7%)
Patients with Hypertension and proteinuria (ACR>30) on angiotensin blockade*	1018(100%)	1073(100%)	883(100%)	190(100%)	135(100%)

a Patients with two consecutive eGFRS under 60 at least seven days apart.

b Patients with a QOF business Rule Read code for CKD.

c Patients with two consecutive eGFRS under 60 at least seven days apart and a QOF business rule Read code.

d Patients with a QOF business Rule Read code for CKD but no sustained eGFRs below 60.

e Patients with two consecutive eGFRS under 60 at least seven days apart but no QOF business Rule Read code for CKD.

Proportions quoted are of the total in that group.

*When comparing groups d and e/c and e, p<0.0001.

+ QOF pay for performance business rules look back 15 months hence time period.

#### Sensitivity Analysis including calculated eGFR from serum creatinine

Inclusion of patients with stages 3–5 CKD calculated from two consecutive serum creatinine results seven days apart gave an adult adjusted prevalence of 4.05% (95% CI 4.03 to 4.10%) in 2005 and 4.66% (95% CI 4.64 to 4.69%) in 2009, peaking at 5.00% (95% CI 4.97 to 5.02%) in 2007. [Figure 3].

**Figure 3:** Prevalence of CKD by year combining CKD stage derived from laboratory eGFRs and eGFR calculated from serum creatinine.

## Discussion

This large primary care based database study has found evidence that the current management of stages 3–5 CKD in UK primary care is systemically suboptimal. Major misclassification of individuals with stages 3–5 CKD was found including both inappropriate labelling as stages 3–5 CKD of those without evidence of stages 3–5 CKD and no labelling of stages 3–5 CKD of others with clear evidence of a reduced eGFR. The finding of an age adjusted prevalence of stages 3–5 CKD in the UK by laboratory reported estimated GFR of 4% in 2008–9, using a definition requiring a confirmed reduction in eGFR to <60 ml/min/1.73 m^2^, was lower than most previous UK primary care estimates of between 4.1 and 8.5% which included patients classified on the basis of a single available eGFR [10], [11], [20], [27].

In patients with stages 3–5 CKD, exclusion from the practice CKD register (‘uncoded’ CKD), was associated with decreasing age, female gender, less co-morbidity (with the exception of hypercholesterolaemia) and lower CKD stage. When comparing uncoded patients with miscoded patients, uncoded patients were less likely to have cardiovascular disease and diabetes but more likely to have hypertension, be older and smoke.

The widespread misclassification shown by this study is important: individuals without an appropriate Read code, despite increased co-morbidity, were less likely to have received adequate care as defined by UK pay for performance targets. Comparison of outcomes for two cardiovascular risk factors (blood pressure and cholesterol) provides some evidence that clinical coding mediates performance for QOF P4P indicators. Uncoded stages 3–5 CKD patients had worse blood pressure control (included in QOF) but similar cholesterol levels (not in QOF) in comparison to miscoded stages 3–5 CKD patients. This also suggests an inappropriate targeting of resources away from individuals in need which could be reversed by better identification of stages 3–5 CKD without increasing workload.

In the sensitivity analysis where patients with either two lab eGFRs or two calculated eGFRs were included the prevalence in 2009 varied from 4% to 4.7%. This suggests a further potential cause of misclassification where laboratory reported eGFR is not available.

### Strengths and Limitations

This is the largest UK cohort study to date to examine stages 3–5 CKD prevalence and comprised approximately 4% of the total UK population. Accounting for the chronicity of stages 3–5 CKD by using two laboratory results rather than a single point estimate has allowed the true burden of stages 3–5 CKD to be more clearly estimated. Although the study aimed to capture stages 3–5 CKD patients diagnosed according to the QOF guidelines, by 2009 the majority of patients diagnosed with stages 3–5 CKD would meet the KDIGO/KDOQI guidelines with lab eGFRs over 90 days apart. It is however possible that some patients who met the QOF guidelines for CKD in fact had acute kidney injury hence did not have CKD on two samples more than three months apart and these would have been incorrectly categorised as miscoded by our study. The methodology differs from other studies by reporting stages 3–5 CKD stages using laboratory reported eGFR, thereby reducing the variation of calculated eGFR due to different creatinine assays [1].

In this study we have performed a multivariable model with a random effects term for primary care practice location, to determine which factors are independently associated with exclusion from the practice register. This model is the most favourable as it takes into account clustering at the practice level.

A limitation of the use of routine data is that 77% of the population did not have two consecutive lab eGFRs reported in the study period. This is likely to result in over-representation of patients with increased co-morbidity (who will have more kidney function tests) and therefore have a higher risk of stages 3–5 CKD. Conversely, it is likely that some individuals with stages 3–5 CKD will not have undergone testing during the time period of the study; however most of the risk factors for CKD (e.g. hypertension, diabetes) are also conditions where routine blood testing is common therefore the majority with stage 3–5 CKD should have been captured.

Ethnicity was not satisfactorily reported in the THIN database and therefore eGFR could not be adjusted for those of black ethnicity. Whilst this could theoretically lead to over-reporting of stages 3–5 CKD prevalence, individuals of black ethnicity only comprise 3.3% of the United Kingdom population so the effect of this limitation should be small [28]. When undertaking the sensitivity analysis there were limitations in calculating the eGFR. The method of creatinine analysis used in the laboratories contributing data to this cohort was not known and therefore analysis did not incorporate the IDMS method as this was not in widespread use during the time period of this study. Prevalence using both serum creatinine and laboratory eGFR appeared to rise and fall over time; this may have been due to changes in the number of laboratories analysing creatinine with the IDMS method.

Laboratory eGFRs and creatinines that were utilised for stages 3–5 CKD prevalence estimates in this study were derived directly from data that were downloaded into the primary care record. Whilst this is complete for patients who had their laboratory tests done from primary care, some patients who were under follow-up in secondary care CKD clinics may not have had their results available. This may have impacted on the prevalence estimates of patients with stage 4 CKD and stage 5 CKD, many of whom are under secondary care follow-up, explaining rates (0.21%) below those reported in other studies.

Finally, it is plausible that GPs may calculate the eGFR themselves and place patients on the CKD practice register. However the GP would have to do this manually as the Vision electronic patient record does not automatically perform this function hence this seems unlikely to have happened on a large scale. Furthermore, this does not explain the issue of uncoded patients and the sensitivity analyses showed that relatively few (0.7%) patients would have been reclassified as stages 3–5 CKD had physicians calculated eGFR themselves. This would therefore not explain the observed miscoding.

### Comparison to the literature

The prevalence estimates for stages 3–5 CKD in this study, with 3.1% of men and 4.8% women affected, were lower than other UK based studies (Appendix A). However the current results were based on two contemporary laboratory reported eGFRs whereas most other UK studies have used a single renal function test to calculate eGFR and therefore have the potential for bias [20], [29]–[31]. Two previous studies need special mention: the QICKD study which included two eGFRs where available and the Health Survey of England which used a single measurement but screened its population [11], [21].

QICKD estimated the “headline” prevalence of stages 3–5 CKD to be 6.8% in a large primary care population but 25% of those labelled as stages 3–5 CKD only had a single eGFR and the study combined laboratory and externally calculated eGFRs. If those with only one eGFR were excluded the prevalence dropped to approximately 5% or under 3% if only laboratory eGFRs were included.

The Health Survey of England Screening study (HSE), using a single eGFR result, reported the prevalence of stages 3–5 CKD as 5% in Men and 7% in women and found the overall prevalence to be 6% [21]. This was a higher proportion than other larger international screening studies which found prevalences of 3.8% (United States) and 4.7% (Norway) also on the basis of a single eGFR [32], [33]. All three of these screening studies are therefore likely to have overestimated the prevalence of stages 3–5 CKD which arguably requires two laboratory eGFRs and a minimum time period between these, as in the KDOQI definition (3 months) or the current study (at least 7 days) [7].

A relationship between increased co-morbidity and appropriate labelling is potentially important, particularly as early CKD may not be associated with higher mortality in otherwise well older people, unlike younger individuals [34]–[36]. The multivariate model in this paper builds on a previous analysis that looked at primary care practitioners in other UK cities. This study showed increasing co-morbidity, age and deprivation at practice level were associated with QOF CKD recording. The current work expands this to individual patients with stage 3–5 CKD: age, male gender, increasing CKD stage, cardiovascular disease and peripheral vascular disease are all associated with appropriate coding [37].

### Clinical Implications

These results suggest that the mechanism for recording stages 3–5 CKD prevalence in primary care needs re-evaluation: relying on manual coding of CKD appears to have resulted in significant misclassification with under treatment of those uncoded and potentially inappropriate intervention in those miscoded. This is consistent with results from a study in Type II diabetes which showed higher HbA1_c_ and worse cholesterol control in patients with diabetes not on the QOF diabetes register [17]. Furthermore, almost twice as many were miscoded as uncoded meaning that improving the accuracy of CKD classification might also reduce workload. One solution for this would be automatic coding on the basis of eGFR results to highlight those at higher risk and similar reclassification of those apparently mislabelled.

These findings may also have implications for estimates of CKD resource use. A recent paper modelled the costs of CKD suggesting these comprised 1.3% of the NHS budget [5]. However this may be an over estimation as some of the costs are based systematically miscoded individuals as seen here [5].

## Conclusions

In summary this paper has shown that robust estimation of the prevalence of stage 3–5 CKD results in generally lower prevalence than previously reported but more importantly uncovers significant misclassification and subsequent sub optimal management of chronic kidney disease. Definitive estimates of prevalence await ongoing screening studies. In the meantime, Primary Care physicians should consider the use of automatic methods to re-classify their CKD population as this may lead to both improved outcomes for patients and reduced workload for primary care practitioners.
